The article "Enterprise Human Resource Optimization Algorithm Using PSO Model in Big Data and Complex Environment" was retracted in 2023. Reasons: signs of a paper mill; suspected computer-generated content; unreliable results or conclusions; concerns about the data.

# Enterprise Human Resource Optimization Algorithm Using PSO Model in Big Data and Complex Environment

**DOI:** 10.1155/2022/1244660

**Published:** 2022-08-31

**Authors:** Xiang Wang, Ying Zhang

**Affiliations:** ^1^College of Political Science and Law, Jiangxi Normal University, Jiangxi, Nanchang 330000, China; ^2^Training Center, Jiangxi College of Foreign Studies, Jiangxi, Nanchang 330000, China

## Abstract

The distribution of human resources has a direct impact on the HR utilization rate in businesses, which in turn has an impact on the profitability and labor productivity of those businesses. As a result, this article develops an enterprise HR optimal allocation model based on PSO. The concepts of HR and HR allocation are introduced, and a programme for implementing optimal HR allocation in businesses is provided from the perspectives of scale prediction, structure analysis, and implementation. An HR configuration optimization model is established, providing a specific method of quantitative management for HR configuration optimization, at the same time starting from operability, based on the methods of system analysis and quantitative evaluation, and an improved PSO is created to address this issue. Results from numerical simulations demonstrate this algorithm's effectiveness. According to the experimental findings, the improved PSO has a quick convergence rate and a roughly 5% lower average error rate than the conventional algorithm. Moreover, this algorithm's accuracy is roughly 94%. This method offers some targeted tactics for optimizing HR configuration.

## 1. Introduction

The process of allocating resources to each project or business unit to maximize profits or reduce costs is referred to as a resource allocation problem. To achieve goal optimization, the primary research challenge in resource allocation is to identify an allocation strategy that can distribute finite resources among a number of tasks while also taking into account resource constraints. The allocation of HR (human resources) is not only the beginning of HRM (human resource management), but it is also the conclusion of HRM [1]. It is the most dynamic factor among the factors affecting human productivity. Its ultimate objective is to match “person-posts” and increase the organization's general effectiveness. Due to the high-tech industries' explosive growth, knowledge-based industries have gradually taken over as society's leading sectors in the era of the knowledge economy, and the employment share of industries that rely heavily on technology and intelligence has significantly increased. Talent has emerged as the “first resource,” and its quantity and quality are the primary drivers of social and economic development [2]. The market competition will shift from the competition of materialised resources like funds and products to the competition of intellectual resources. The competition between enterprises is essentially the competition of talents. To improve their competitive ability in the fierce market competition, enterprises must strengthen the integration and application of their own resources [3]. If the allocation of HR in an enterprise is unreasonable, there will be ups and downs in HR usage. In the peak period of resource utilization, the maximum HR demand in some time periods will exceed the HR limit in that time period, which will cause the work to be unable to proceed normally and, at the same time, increase the load of the support system and affect the quality of support [4]. In a period of low resource utilization, problems such as underutilization of HR will affect the coordinated management of technical support. The efficiency of HR allocation will directly affect the utilization rate of enterprise HR and then affect the labor productivity and economic benefits of the enterprise. Therefore, the research on the optimal allocation of enterprise HR has certain practical significance.

PSO (particle swarm optimization) is an evolutionary algorithm based on swarms that mimics the foraging behaviour of birds in flight and accomplishes the best outcome by relying on the group cooperation of the birds [5]. A mechanism exists for the entire flock of birds to communicate with one another while they are foraging. The flock's consistency in the foraging process is ensured by their constant changes in flight direction and good spacing between individuals. This is a wise action to take. Every PSO particle is a solution in the solution space, and each one adjusts its flight in accordance with its own flight experience and the experiences of its companions [6]. Each particle state in the algorithm's search space represents a potential answer to the optimization conundrum and a fitness value assigned by the target objective function. The basic PSO can only look for one extreme point uncertainly at a time [7]. The fundamental PSO is inappropriate for multimodal optimization issues because of these features. Additionally, the basic PSO has poor convergence accuracy and is prone to local optimum, which prevents the algorithm's optimization effect from reaching its full potential. This study enhances the fundamental PSO. Because there are currently no effective scientific methods for allocating personnel, the desired outcome is frequently not realized. Therefore, this article establishes an enterprise HR optimal allocation model based on PSO, which better meets the needs of system optimization in HR optimal allocation through the discussion and analysis of HR optimal allocation. The following are its innovations:

1. This article introduces the concepts of HR and HR allocation and gives the program of HR optimal allocation in enterprises from the aspects of scale prediction, structure analysis, and implementation. At the same time, in order to improve the utilization efficiency of HR resources, this article studies the optimization method of HR allocation. The results show that this method provides countermeasures and ideas for realizing HR allocation optimization in enterprises.
2. Combining theory, model, and demonstration, this article constructs the research system of HR allocation optimization in enterprises and gives the methods, objectives, and countermeasures of HR allocation optimization. At the same time, in order to make the optimization algorithm search the area where the extremum is located more carefully, this article proposes a fitness distance similarity model and a new adaptive multimodal PSO based on this similarity model. The results verify the feasibility and effectiveness of this method in HR configuration optimization.

This article mainly explores the optimal allocation of HR in enterprises. The article is divided into five section, and the specific research framework is as follows: Section 1 is the introduction. This part mainly expounds the research background and significance of the article, analyzes the research status of HR optimal allocation in enterprises, and puts forward the research purpose and content of this article. Section 2 mainly summarizes and studies the related literature and introduces the research methods of this article. Section 3 is the method part, focusing on the construction method and implementation of enterprise HR optimal allocation model based on PSO. Section 4 is the experimental analysis. In this part, experiments are carried out on data sets to analyze the performance of the model. Section 5 presents the conclusion and prospect. This part mainly reviews the main contents and results of this research, summarizes the research conclusions, and points out the direction of further research.

## 2. Related Work

Mahdjouba and Nasreddine embedded the idea of the genetic algorithm into PSO according to the characteristics of the mathematical model of HR optimal configuration and designed an improved PSO to solve this problem. The numerical simulation results show the effectiveness of the algorithm [8]. Michael et al. took temporal database theory as the basic theory, combined personnel information with file management, combined basic information with derived information, static information. and dynamic information to form an integrated data source. They constructed a distributed HRM information system [9]. Nishino et al. studied the evaluation model of the resource balance optimization problem. The model introduces an optimization method based on dynamic time difference; proposes a resource balancing optimization method based on PSO; selects an example to conduct an example verification, which verifies the effectiveness of the method [10]. Liu et al. pointed out that, in order to ensure the scientificity and fairness of the score, when evaluating and scoring personnel, it is generally necessary to consider various scoring factors and their respective weights in the scoring [11]. Luo proposed a HR configuration method based on a multiobjective hybrid genetic algorithm. That is, a multistage decision-making model is used to deal with this problem, and the task is regarded as a series of interactions between the decision-maker and the outside world. There are some available decisions in each stage, and their immediate effects can be easily calculated [12]. Sena et al. analyzed the main problems existing in the HR allocation of state-owned enterprises by discussing the internal and external conditions of HR allocation of state-owned enterprises [13]. Aiming at the problem that the actual scheduling process is constrained by multiple resources, Nadkarni and Stening established a dual-resource multiobjective scheduling model considering the differential operation efficiency [14]. Based on the idea of system science, Beal and Astakhova conducted an in-depth analysis of the problems existing in HR planning at this stage and constructed a model library of enterprise HR planning [15]. Haworth built an HRM system based on a temporal data model. The feature of this system is that it is based on components and conforms to national standards, so each module is easy to flexibly expand and combine according to the actual situation and has universality [16]. Zhu and Verstraeten gave the grey system model, production function model, and multiple linear regression model for predicting the scale of enterprise HR optimized configuration and proposed a forecasting method to select three satisfactory models from a number of models that passed statistical tests to determine the combination; four methods for determining the combined weights are given [17]. Taking the configuration problem of enterprise HR as the research object, Li and Sun chose the principal component analysis method to evaluate the configuration efficiency of enterprise HR [18]. Schirmer and Drexl constructed an enterprise HR configuration efficiency index system from five aspects: quantity configuration, structural configuration, quality configuration, benefit, and cost based on the related theory of HR configuration [19].

Based on the research on the optimal allocation of enterprise HR in related literature, this article puts forward a new research perspective and method. In this article, the concepts of HR and HR allocation are introduced, and the procedures of HR optimal allocation in enterprises are given from the aspects of scale prediction, structure analysis, and implementation. At the same time, in order to make the optimization algorithm search the area where the extremum is located more carefully, this article proposes a fitness distance similarity model and a new adaptive multimodal PSO based on this similarity model. The results verify the feasibility and effectiveness of this method in HR configuration optimization. This article provides countermeasures and ideas for realizing HR allocation optimization in enterprises.

## 3. Methodology

### 3.1. Related Theoretical and Technical Basis

HR allocation mainly studies the allocation of HR quantity, quality, and structure in enterprises. Quantity, mainly to study whether the existing HR quantity matches the required quantity of the enterprise's production and operation, refers to the education level and training status of the existing HR, and the key is the structure of knowledge and working ability, mainly to study whether the enterprise HR collocation is reasonable and efficient. The key factors affecting the competitiveness of enterprises are the unique HR and intellectual capital of enterprises, which are directly related to the survival and development of enterprises. After the managers realized the importance of HR, the HRM work within the enterprise has also become an important job in the enterprise, and its position has been upgraded from tactical level to strategic level. Nowadays, the HRM department has changed from the original role of administration, general affairs, and welfare committee to the strategic business partner of the enterprise, the consultant of senior executives, the promoter of education, and the advocate of change. HRM has changed from transactional management to strategic HRM. The quality of HR is a comprehensive indicator of the quality of labor force, and it is the knowledge, wisdom, skill level, and labor attitude that HR possesses. It is embodied in workers' physique level, professional and technical level, knowledge and culture level, labor enthusiasm, etc. It is a measurable index. The matching between HR allocation and enterprise strategy is intended to establish an extremely effective HRM mechanism and enhance the competitive soft power of enterprises. Matching or not is the key to affecting enterprise performance and solid support to achieve enterprise strategic goals. HR configuration has the following characteristics: (1) the object of HR configuration has initiative. As an object of HR allocation, although it exists as the object of HR allocation, the object itself is dynamic. (2) HR configuration is bidirectional. The configuration of HR is two-way. Both the subject and the object of the configuration are human beings, and they all have subjective initiative.

Any organization is a system. What kind of people need to be assigned to a specific position should be designed according to the overall optimization of the system, rather than just selecting the best employees in the same position. This means that when selecting personnel, there should be a good process of identification and selection, and the needs of having the corresponding skills, knowledge, and experience and realizing the optimization of the organizational system should be selected. The macroallocation of HR refers to the allocation of HR in a country. Microallocation of HR refers to the scientific and rational allocation of HR within a specific organizational system. Of course, microallocation involves many problems, such as organization setup, management level, management range, work design, operation mechanism, management mode, and staff quality. The technical path dependence of HRM must change along with the change in HRM's role. Development and use of information system technology have evolved into a crucial and essential link in the chain-type HR configuration optimization activities in order to avoid organizational information distortion and the internal friction of delayed information. At the moment, the combination explosion of the search will happen if we cannot use the inherent knowledge of the problem to narrow the search space. The general search algorithm to find the optimal or nearly optimal solution is thus a fascinating topic because research can automatically acquire and accumulate knowledge about the search space in the search process and control the search process adaptively. The benefits of PSO are its ease of use, quick convergence, and the limited number of parameters that need to be changed. Currently, this algorithm is frequently used in application areas such as function optimization, neural network training, pattern classification [20], and fuzzy system control. PSO, however, has its own drawbacks. For instance, an algorithm's iterative process depends on the value of its parameters, but choosing the right parameters can be challenging. Different models require different parameter choices. The algorithm quickly converges in the early stages of optimization, but the final result is not optimal and there is no reliable method of causing the algorithm to depart from the minimum point [21]. The initialization phase and the postevolution process of the particle swarm are improved in this article when using PSO to solve the problem, preventing the calculation from reaching an infeasible solution. The PSO process is shown in Figure 1.

When compared to other economic resources, human resources are clearly cyclical and unsustainable. The overall HR function can be strengthened by effective HR allocation, which also aligns people's skills with job demands. By projecting future internal HR demand and supply for businesses, HR planning can identify the difference between supply and demand. At this point, the definition of the HR planning concept completes its information. It primarily consists of five components: setting enterprise goals, creating enterprise plans, forecasting internal demand for HR, analyzing internal employee characteristics, forecasting internal supply, calculating net demand for HR, and creating plans to ensure the balance of internal supply and demand for HR. A portion of the work done to create a rational enterprise HR plan ensures that resources are used in a balanced manner, reducing fluctuations in HR demand during use, making scheduling management easier, and increasing resource utilization. This is the optimal HR allocation in the enterprise problem. The actual optimal HR allocation requires that it be chosen and distributed in accordance with the unique organizational structure situation and the position's emphasis on the skill requirements of the workforce. The weighting of each competency element in various positions, as well as the candidates' scores on the various competency elements required by their positions, must typically be taken into account. The distribution of HR is more rational and scientific, and the creation of a good system encourages employee enthusiasm and creativity, enhancing organizational and work efficiency. The fundamental tenets of resource allocation, which apply to HR as well, are scientific forecasting, allocation optimization, and realizing the scientific combination of people and things. The most effective HR resource allocation in an organization not only increases internal HR's utilization rate but also serves as a crucial foundation for HRM training, promotion, and recruitment.

### 3.2. Establishment of the HR Optimal Allocation Model in Enterprises

The external environment of enterprises that affects HR demand mainly includes social and economic environment, social, political, legal, and other factors, technological change, and technological innovation. The internal factors of an enterprise, including the overall development strategy, the business scope, the adjustment of the enterprise structure, and the financial budget of the enterprise, will all affect the HR demand of the enterprise. At the same time, according to the concepts of HR allocation and HR allocation efficiency, the factors that determine the HR allocation efficiency of an enterprise include five aspects: quantity allocation, structure allocation, quality allocation, revenue, and cost. In this article, the original collected and irregular data are processed to make it regular and regular to follow, instead of directly using the original data to model and then using the generated regular data columns to analyze and model. HR information is the basis of HR configuration optimization. In the HRM of the whole enterprise, the role of information runs through the process from forecasting and decision-making to planning, organizing and implementing, and controlling. Whether the forecast is accurate and the decision is scientific is related to the survival and development of enterprises. Whether the HR allocation of an enterprise has reached the most effective level will directly affect the realization of the enterprise's business objectives and maximum benefits. When the efficiency of HR allocation is high, the utilization rate of HR will be enhanced and the enterprise benefit will be improved. Because different positions have different responsibilities and different requirements for personnel's ability, it is necessary to determine the weight distribution of various ability elements in each position. According to the relative importance of elements, the 9-scale method can be used to compare various elements, and the judgment matrix can be obtained. Then, the weight vector is obtained by calculating the maximum eigenvalue of the judgment matrix by AHP. The enterprise HR configuration scheduling process is shown in Figure 2.

By analyzing the composition and structure of the particle swarm, we can know that the first part is the velocity of particles, which represents the velocity of the previous state of particles, and it reflects the current state, which plays a role in grasping the global and local search. Secondly, the middle part is the part where the particles learn by themselves. The particles search for their own optimal value, which enhances their global search ability and avoids falling into local extremum. The last part is the social part, in which particles approach the global optimal value, representing the cooperation and information sharing among particles. In this article, the update speed of parasitic swarm particles is updated by elite learning strategy, and the speed of host swarm particles is updated by compression factor PSO. The rule of the evaluation function is that the smaller the mean square error of resource usage, the larger the individual fitness value. With the evolution of particle swarm, “the algorithm finally finds the resource plan with the smallest variance.” Therefore, the original objective function should be converted into a fitness value function to ensure that the suitable individual has a large fitness value. When the number of people and posts involved is relatively small, it can be solved by the Hungarian method. However, when the number of people and posts involved in the problem is large, the problem becomes more complicated. An improved PSO is designed to solve this problem. In this article, a fitness distance similarity model is proposed, and a new adaptive multimodal PSO is proposed based on this similarity model. The biggest difference between this algorithm and other multimodal optimization algorithms is that it does not need to set any parameters related to specific problems.

In the mathematical model of the dual-criteria HR optimal allocation problem, *M* employees are allocated to *n* different projects to maximize profits and minimize costs under resource constraints. It is represented as a bicriteria integer programming model as follows:

(1) $$\begin{array}{c} \text{Max}z_{1}\left(y\right)=\overset{n}{\underset{i=1}{\sum }}f_{1}\left(y_{i}\right),\\ \text{Min}z_{2}\left(y\right)=\overset{n}{\underset{i=1}{\sum }}f_{2}\left(y_{i}\right),\\ s.t.G_{0}\left(y\right)=\overset{n}{\underset{i=1}{\sum }}g_{i}\left(y_{i}\right)\leq M,\\ y_{i}=0,1,2,3,\ldots ,M\forall i,\\ i=\left(1,2,3,\ldots ,N\right)\;j=\left(1,2,3,\ldots ,M\right). \end{array}$$

Among them, *i* refers to the enterprise project index; *j* refers to the enterprise employee index; *N* refers to the total number of enterprise projects; *M* refers to the total number of enterprise employees. Let the vector of each particle be

(2) $$\begin{array}{c} X=\left(x_{1},x_{2},x_{3},\ldots ,x_{i},\ldots ,x_{n}\right). \end{array}$$

It means that personnel *i* are assigned to post *x*_*i*_, where

(3) $$\begin{array}{c} i=1,2,3,\ldots ,n\;x_{i}\neq x_{j}\left(i\neq j\right). \end{array}$$

In this article, the index of mean square error *σ*^2^ is used to judge the balance of resource demand; that is, the dispersion degree of resource consumption per unit time from the horizontal line *y*=*Q*_*m*_ is used to measure the pros and cons of a scheduling scheme. The ideal situation is that the resource dynamic curve is close to a rectangular distribution, that is, a rectangle with *Q*_*m*_ as the height and the specified construction period as *T* as the length. The model for resource balancing optimization is as follows:

(4) $$\begin{array}{c} \text{Min}E=\frac{1}{T}\int_{0}^{T}{\left[R\left(t\right)-R_{m}\right]}^{2}\text{d}t=\frac{1}{T}\int_{0}^{T}R^{2}\left(t\right)\text{d}t-R^{2}{}_{m}\circ s.\mathrm{t.},\\ R\left(t\right)=\sum_{\left(i,j\right)}R_{i,j}\left(t\right)\left(i,j\right)\in W,\\ R_{i,j}\left(t\right)=\left\{\begin{array}{cc} R_{i,j}^{0}t_{A}, & \left(i,j\right)\leq t\leq t_{A}\left(i,j\right)+d\left(i,j\right),\\ 0, & \text{else}, \end{array}\right.\\ t_{A}\left(k,i\right)+d\left(k,i\right)\leq t_{A}\left(i,j\right)\left(k,i\right)\in F\left(i,j\right),\\ t_{ES}\left(i,j\right)\leq t_{A}\left(i,j\right)\leq t_{LS}\left(i,j\right), \end{array}$$

where *T* is the total duration of the task and *A* is the fixed value; *R*(*t*) is the sum of resource consumption of all work in the *t* time unit; *R*_*m*_ is the average value of the current network plan resource intensity distribution; *R*_*i*,*j*_(*t*) is the resource intensity of working (*i*, *j*) at *t* time; *t*_*ES*_(*i*, *j*) is the earliest commencement time of (*i*, *j*); *t*_*LS*_(*i*, *j*) is the latest commencement time of (*i*, *j*); *t*_*A*_(*i*, *j*) is the actual commencement time of (*i*, *j*); *d*(*i*, *j*) is the duration of working (*i*, *j*); *F*(*i*, *j*) is the collection of all emergency work of working (*i*, *j*). The model has *p* objectives, namely,

(5) $$\begin{array}{c} f_{1}\left(x\right),f_{2}\left(x\right),f_{3}\left(x\right),\ldots ,f_{p}\left(x\right). \end{array}$$

Among them, *x* ∈ *R*^*n*^ is a vector or *n* decision variables.

Comprehensive, accurate, and timely information is the premise and basis of scientific decision-making. Therefore, the information work of enterprise personnel management is the basic work of enterprise personnel management. Numerous, accurate, multidimensional, and frequently updated personnel data are available. The initialization of the particle swarm must be adjusted because the total time difference of the activities is dynamic. In addition to determining the spatial coordinates of the particle with the longest actual completion time among all of the activity's immediate predecessors, it is necessary to determine whether the activity corresponding to a particular dimension of each particle has an immediate preceding activity. The relationship between input and output is described mathematically using the production function model. It is used to forecast the allocation of HR scale development trends. This is due to the interactions between an organization's HR, business operations, and production. The initialized position vector is mapped to the weights and thresholds of the network by the input training sample as the current global optimal value. The mean square error between the expected and actual output is calculated, and it is used as the fitness function for PSO. The initialization of the particle swarm and the postevolution of the particle swarm processes in this article make sure that each particle's position is always within the feasible solution space and that the generated solution always solves the intended problem, preventing the generation of infeasible solutions.

## 4. Result Analysis and Discussion

PSO seeks the optimal solution through the cooperation between individuals, and its essence is to use the information of individual extremum and all extremum to guide the next iteration of particles. In this article, an improved PSO is proposed to solve the problem of HR optimal allocation. In order to verify the feasibility and reliability of this method, experiments are carried out in this section. In this section, enterprise A is taken as the object, and the simulation experiment is carried out. In order to make the results more in line with the objective reality, recent data are selected to determine the optimal allocation target of the enterprise HR scale. Therefore, this article selects the data from 2010 to 2015 and uses the improved PSO method to determine the optimal allocation target for enterprise HR scale. The raw data of HR scale allocation of enterprise A from 2010 to 2015 and the cumulative processing data are shown in Table 1.

Let the particles in the current particle swarm cross-operate with all the optimal particles first, select the offspring individuals with high fitness value, and then cross-operate with the individual optimal particles, take the offspring individuals with high fitness value as new particles, and iterate in turn until the iteration termination condition is met. At this time, the optimal particle in the particle swarm is the optimal solution. Firstly, the algorithm experiments are carried out many times, and the convergence rate of the algorithm is shown in Figure 3.

The quantity allocation efficiency of HR owned by an enterprise is the guarantee for an enterprise to improve its HR allocation efficiency. Only when an enterprise has the total amount of HR that adapts to the development of the enterprise, can it effectively allocate the HR of the enterprise according to the enterprise's production and management objectives and the needs of the enterprise's production and sales. The efficiency of HR configuration optimization using different methods is shown in Figure 4.

Experiments show that the optimization algorithm proposed in this article can get the optimal solution to the problem quickly, and it has obvious advantages in the case of more personnel and posts and improves the efficiency of personnel allocation. It is an effective algorithm to solve the HR optimal allocation problem. Comparing the average error rates of different algorithms, the results are shown in Figure 5.

It can be seen from Figure 5 that with the increase of evolutionary algebra, the average error rate of each algorithm is constantly decreasing and finally tends to be stable. However, the average error rate of this article is the smallest, which shows that the performance of this model is better.

The unmodified PSO and the improved PSO are used to solve the HR allocation problem, respectively. The comparison between the algorithm before and after improvement is shown in Figure 6.

According to the characteristics of each post, determine the evaluation method of personnel quality or build a competency model in the process of measures implementation so as to inspect personnel quality, and ensure the implementation of HR plan by making HR training plan, personnel recruitment plan, HR use, and deployment plan.

Decision-makers must identify the best HR allocation path with double criteria when solving the double-criteria HR allocation problem in multistage combinatorial optimization problems. The number of function evaluations is the primary calculation expense when solving multimodal optimization problems. As a result, by calculating the function's evaluation times, the calculation cost of the algorithm can be determined. The calculation cost of an optimization algorithm is relatively low if it requires fewer function calls than other optimization algorithms, which indicates better performance. The precision comparison of different algorithms is shown in Figure 7.

Forecasting the HR demand of enterprises can help enterprises to make clear the future HR demand trend, avoid the loss caused by excessive demand and waste of personnel, improve the efficiency of HR recruitment, avoid the shortage of HR, and guide HR training, thereby improving the HR allocation efficiency, further maintaining the stable operation of enterprises, preventing business risks, and maximizing the benefits of enterprises. The comparison between the calculated results of this model and the actual values is shown in Table 2.

It can be seen that the actual value is close to the model analysis value. This shows that using this method to predict the development trend of enterprise HR allocation has a good effect.

The experimental results in this section show that the improved PSO has a fast convergence speed, and the average error rate of the improved PSO is about 5% lower than that of the traditional algorithm. And the accuracy of this algorithm is about 94%. In this section, the method has solved the problem of personnel optimal allocation when there are a large number of personnel and posts and it improved the efficiency of personnel allocation.

## 5. Conclusions

The first resource for advancing technology and business growth, HR has evolved into a science. One of these is the study of HR optimal allocation, which is a key component of HR strategic management. The effectiveness of HR allocation will have a direct impact on the economic advantages and labor productivity of businesses. As a result, HR allocation plays a crucial role throughout the enterprise management process. This article establishes a mathematical model of HR optimal allocation through discussion and analysis of HR optimal allocation, which better satisfies the requirements of system optimization in HR optimal allocation. Additionally, this article suggests a fitness distance similarity model and a new adaptive multimodal PSO based on this similarity model to help the optimization algorithm search the region where the extremum is located more carefully. According to the experimental results, the improved PSO has a quick convergence rate and a roughly 5% lower average error rate than the conventional algorithm. And this algorithm's accuracy is around 94%. The outcomes demonstrate the viability and efficacy of the HR configuration optimization approach presented in this article, and the algorithm exhibits undeniable superior performance. The method described in this article simultaneously increases the effectiveness of personnel allocation while resolving the issue of personnel optimal allocation under conditions of high personnel and postdensities. There are still some areas where the research process needs to be improved, even though this article has made some research advancements on the optimal allocation of HR in enterprises. This article does not conduct a thorough investigation into the effectiveness of HR. According to the HR circumstances and job characteristics of a particular enterprise, we can determine the necessary quality requirements and HR characteristics in practice. As a result, more research is needed on the HR quality model.

## Figures and Tables

**Figure 1:** PSO process.

**Figure 2:** Enterprise configuration scheduling process.

**Figure 3:** Convergence rate of the algorithm.

**Figure 4:** Efficiency comparison of HR configuration optimization.

**Figure 5:** Average error rate of algorithm.

**Figure 6:** Comparison of the algorithm before and after improvement.

**Figure 7:** Comparison of the accuracy of the algorithm.

**Table 1:** 2010–2015 HR scale allocation table of enterprise A.

Age	2010	2012	2013	2014	2015	2016
Employee scale	1865	1811	1742	1653	1534	1327
x^(0)^ (i)	x^(0)^ (1)	x^(0)^ (2)	x^(0)^ (3)	x^(0)^ (4)	x^(0)^ (5)	x^(0)^ (6)

**Table 2:** Comparison between calculated results and actual values by model analysis.

Index	2010	2012	2013	2014	2015	2016
Actual value	1865	1811	1742	1653	1534	1327
Model analysis value	1885	1798	1703	1634	1489	1299

## Data Availability

The data used to support the findings of this study are available from the corresponding author upon request.
